# Identification of Therapeutic Targets and Prognostic Biomarkers among Genes from the Mediator Complex Family in the Hepatocellular Carcinoma Tumour-Immune Microenvironment

This article has been retracted.

**DOI:** 10.1155/2022/2021613

**Published:** 2022-01-13

**Authors:** Wei Tan, Shuai Peng, Zhuokai Li, Ruiqian Zhang, Yangrui Xiao, Xiao Chen, Jinde Zhu, Bingrong Li, Xinliang Lv

**Affiliations:** ^1^Department of Hepatobiliary and Pancreatic Surgery, Lishui Central Hospital, Fifth Affiliated Hospital of Wenzhou Medical College, Lishui City, Zhejiang Province 323000, China; ^2^Department of Radiology, The First Affiliated Hospital of Guangxi Medical University, Nanning City, Guangxi Zhuang Autonomous Region 530021, China; ^3^Department of Radiology, Lishui Central Hospital, Fifth Affiliated Hospital of Wenzhou Medical College, Lishui City, Zhejiang Province 323000, China

## Abstract

**Background:**

Hepatocellular carcinoma (HCC) is predominant among all types of primary liver cancers characterised by high morbidity and mortality. Genes in the mediator complex (MED) family are engaged in the tumour-immune microenvironment and function as regulatory hubs mediating carcinogenesis and progression across diverse cancer types. Whereas research studies have been conducted to examine the mechanisms in several cancers, studies that systematically focused on the therapeutic and prognostic values of MED in patients with HCC are limited.

**Methods:**

The online databases ONCOMINE, GEPIA, UALCAN, GeneMANIA, cBioPortal, OmicStudio, STING, Metascape, and TIMER were used in this study.

**Results:**

The transcriptional levels of all members of the MED family in HCC presented an aberrant high expression pattern. Significant correlations were found between the MED1, MED6, MED8, MED10, MED12, MED15, MED17, MED19, MED20, MED21, MED22, MED23, MED24, MED25, MED26, and MED27 expression levels and the pathological stage in the patients with HCC. The patients with high expression levels of MED6, MED8, MED10, MED17, MED19, MED20, MED21, MED22, MED24, and MED25 were significantly associated with poor prognosis. Functional enrichment analysis revealed that the members of the MED family were mainly enriched in the nucleobase-containing compound catabolic process, regulation of chromosome organisation, and transcriptional regulation by TP53. Significant correlations were found between the MED6, MED8, MED10, MED17, MED19, MED20, MED21, MED22, MED24, and MED25 expression levels and all types of immune cells (B cells, CD8^+^ T cells, CD4^+^ T cells, macrophages, neutrophils, and dendritic cells). B cells and MED8 were independent predictors of overall survival. We found significant correlations between the somatic copy number alterations of the MED6, MED8, MED10, MED20, MED21, MED22, MED24, and MED25 molecules and the abundance of immune infiltrates.

**Conclusions:**

Our study delineated a thorough landscape to investigate the therapeutic and prognostic potentials of the MED family for HCC cases, which yielded promising results for the development of immunotherapeutic drugs and construction of a prognostic stratification model.

## 1. Introduction

Liver cancer ranked sixth in terms of global incidence and third in all-cause cancer mortality worldwide in 2020 [1]. Hepatocellular carcinoma (HCC) is a predominant type of primary liver cancer. Despite novel therapeutic treatments such as immune therapy, neoadjuvant oncological therapy, and combination therapies parallelly conducted in clinical trials, the 5-year survival rate of HCC remains poor, with an average of <5% [2]. Recently, accumulating evidence has elucidated the pivotal role of the tumour microenvironment in determining tumour-immune interactions, which directly respond to treatment, mediating carcinogenesis and progression [3]. However, the scarcity of efficient therapeutic targets and prognostic biomarkers has limited the patient benefit from novel immune therapies.

The mediator complex (MED) family, consisting of a conserved multiprotein complex ranging from elegans to mammals, interacts with coactivators to direct transcription by RNA polymerase II [4]. Cumulative evidence has shown a close relationship between the MED family and cancer biology, involving EGFR signalling, Wnt signalling, ERK/MAPK signalling, and cell cycle [5]. Aberrant expressions of the members of the MED family have been reported in diverse cancers, indicating their role as a regulatory hub [6–8]. Moreover, members of the MED family have been examined in depth for their protective curative potential for cancers. Specifically, a mechanistic study demonstrated that downregulation of MED19 expression might be a promising treatment approach for inhibiting the cell growth and proliferation potential of breast cancer [9]. In addition, lowering the expression levels of MED1 and MED17 could inhibit proliferation, inhibit the cell cycle, and induce apoptosis in prostate cancer [10]. Recently, fuelled attention has been given to investigations on the response and regulation of the immune system in oncology [11, 12]. With their immune-modulating potential, members of the MED family are promising therapeutic and prognostic biomarkers for different types of cancers.

Whereas research studies have been conducted to examine the mechanisms in several cancers, studies that systemically focused on the therapeutic and prognostic values of the MED family in patients with HCC are limited. As bulk data generated by microarray and sequencing have been shared online, an integrated systemic analysis is possible under the background of precision medicine. In this study, we performed a comprehensive analysis of members of the MED family to elucidate their therapeutic and prognostic potentials. Thereby, we aimed to provide new insights for understanding the mechanisms of members of the MED family that have been implicated in the immune system and a novel treatment option for clinicians to maximise the benefits for patients with HCC.

## 2. Materials and Methods

### 2.1. ONCOMINE

ONCOMINE (http://www.oncomine.org) as a powerful platform with large cancer microarray data has laid a foundation for translational bioinformatics [13]. Data on the expression levels of members of the MED family in HCC were examined using the following conditions: *p* value of 0.05, fold change of 2, and only genes in the top 10% of the data were extracted to evaluate the expression levels of members of the MED family. An analysis was performed using the Student *t* test to compare the discrepancy in the expression level.

### 2.2. UALCAN

UALCAN (http://ualcan.path.uab.edu/analysis.html) is an online web tool that facilitates in-depth analysis with TCGA level 3 RNA-seq and clinical data from 31 cancer types [14]. In the “TCGA gene analysis” module, the expression data of the MED family were analysed using the “liver hepatocellular carcinoma” TCGA dataset. Statistical analysis was performed using a two-tailed Student *t* test, with a cutoff *p* value of <0.05.

### 2.3. GEPIA

The online database GEPIA (http://gepia.cancer-pku.cn/) is a user-friendly, interactive website integrating transcriptome data from the TCGA and GTEx projects for bioinformation analysis [15]. In the “single-gene analysis” module, the correlations between the expression levels of members of the MED family and pathological stage and the prognostic values of the selected genes were investigated. The top 10 most similar genes for each member of interest of the MED family were extracted for subsequent functional analysis. In the “multiple-gene comparison” module, a multiple gene comparison analysis was performed to plot a thorough expression matrix based on a given gene list. The chosen cutoff *p* value was 0.05. The Student *t* test was used for *p* value generation both in the expression and pathological stage analyses. Survival curves were created using the Kaplan-Meier method.

### 2.4. cBioPortal

cBioPortal (http://www.cbioportal.org), characterised with a comprehensive analysis of multidimensional cancer genomic data, provides attractive interactive experiences to examine genetic, epigenetic, transcriptional, and proteomic information [16]. The “mutations” module, which has 373 HCC samples available, was queried to obtain a comprehensive mutation landscape of the members of interest of the MED family in the “liver hepatocellular carcinoma (TCGA, Firehose Legacy)” dataset on the cBioPortal website. Transcriptional data (RNA-Seq V2 RSEM) of the MED family with a *z*-score threshold of ±2.0 were downloaded from cBioPortal for subsequent correlation analysis in OmicStudio.

### 2.5. OmicStudio

OmicStudio (https://www.omicstudio.cn/tool) is an integrated web tool for visualising user-defined data, including genomic, transcriptional (including single-cell analysis), and microbiomic information. Pearson correlation analysis of the MED family was performed using the transcriptional data downloaded from the cBioPortal web tool and visualised in OmicStudio.

### 2.6. STRING

STRING (https://string-db.org/) allows users to perform gene-set enrichment analysis of the entire input with a comprehensive analysis of protein-protein interaction [17]. A protein-protein interaction network was constructed to investigate the interactions of the members of interest of the MED family at the protein level.

### 2.7. GeneMANIA

GeneMANIA (http://www.genemania.org) is a powerful, flexible website for analysing genomic and proteomic information of submitted genes that uses GEO, BioGRID, Pathway Commons, I2D, and organism-specific functional genomic datasets [18]. Protein interaction networks of the MED family were constructed as a supplementary analysis to examine potential interactions with external genes at the protein level by using pathway, physical, and genetic interactions and predicted networks in the online GeneMANIA website.

### 2.8. Metascape

Metascape (http://metascape.org) allows experimental biologists to analyse OMIC-based datasets, providing a one-stop tool for analysing functional enrichment, interactive analysis, gene annotation, and so forth [19]. Gene annotation and functional enrichment analyses of the genes in the MED family and most similar neighbour genes were performed within the “express analysis” module.

### 2.9. TIMER

TIMER (https://cistrome.shinyapps.io/timer/) provides an intuitive web interface for systemically analysing and visualising tumour-immune interactions among 10,897 tumour samples from 32 cancer types [20]. The “gene” module was examined to depict the correlation between MED family members and immune infiltration. The “survival” module was used to analyse the prognostic value of the MED family and determine the independent prognostic predictors. The “SCNA” module was queried to evaluate the correlation between somatic copy number alterations (CNAs) and the abundance of immune infiltrates.

## 3. Results

### 3.1. Expression Patterns of MED Family Members in Patients with HCC

Twenty-nine molecules in the MED family were examined using the online database ONCOMINE. We first qualitatively compared the transcriptional levels of the genes in the MED family in HCC and normal liver tissue specimens (Figure 1). The results showed that only the expression level of MED25 was significantly elevated (*p* = 1.25*E* − 04), while that of MED26 (*p* = 0.037) was significantly reduced at the RNA levels in the HCC and normal liver tissue specimens.

To further test the potential role of the MED family in tumorigenesis and tumour development, we used the UALCAN web tool to quantitatively assess the transcriptional levels of MED family members. As shown in Figure 2, we found that all the molecules in the MED family showed aberrantly high expression patterns in the HCC tumour specimens compared with the normal tissue specimens. Moreover, we showed comprehensive expression patterns of the MED family members. Among the genes in the MED family, MED16 showed the highest relative expression level with a score of 5.2, whereas MED26 scored 2 as the counterpart with the lowest expression level (Figure 3).

We next used GEPIA to study the clinical pathological stage linking all members of the MED family. We found significant correlations between the expression levels of MED1 (*p* = 0.0159), MED6 (*p* = 0.0375), MED8 (*p* = 0.00697), MED10 (*p* = 0.0342), MED12 (*p* = 0.0339), MED15 (*p* = 0.00393), MED17 (*p* = 0.0265), MED19 (*p* = 0.00942), MED20 (*p* = 0.0341), MED21 (*p* = 0.00833), MED22 (*p* = 0.00023), MED23 (*p* = 0.0353), MED24 (*p* = 0.0269), MED25 (*p* = 0.000557), MED26 (*p* = 0.0496), and MED27 (*p* = 0.00569) and the pathological stage (Figure 4). We excluded MED4, MED7, MED9, MED11, MED13, MED14, MED16, MED18, MED28, MED29, MED30, and MED31 from further analysis, as their expression levels were not correlated to the clinical pathological stage. Collectively, these data suggest that the members of the MED family play substantial roles in tumour formation and progression in HCC.

### 3.2. Prognostic Value of the MED Family in Patients with HCC

To investigate the role of the MED family in the progression of HCC, we performed a survival analysis with different end points on the GEPIA website. We first chose overall survival (OS) as the end point event. The patients with HCC who had high expression levels of MED6 (*p* = 0.0043), MED15 (*p* = 0.0039), MED17 (*p* = 0.011), MED19 (*p* = 6.8*E* − 06), MED21 (*p* = 0.042), MED22 (*p* = 0.012), MED24 (*p* = 0.019), and MED25 (*p* = 0.014) were significantly associated with worse overall survival. Moreover, the low expression levels of MED8 (*p* = 0.00012) and MED10 (*p* = 5.4*E* − 05) were significantly associated with longer OS in the 5-year follow-up period, but not in the 10-year follow-up period (Figure 5). Next, we estimated the role of the MED family in prognostic stratification by using disease-free survival (DFS). We found that the high expression levels of MED10 (*p* = 0.04), MED19 (*p* = 0.0057), MED22 (*p* = 0.011), and MED25 (*p* = 0.0019) were significantly associated with worse DFS. Moreover, the low expression levels of MED8 (*p* = 0.027), MED20 (*p* = 0.025), and MED24 (*p* = 0.0027) were significantly associated with longer DFS in the 5-year follow-up period, but the survival benefits had diminished at the 10-year follow-up period (Figure 6). For further analysis, we chose molecules in the MED family that had definite prognostic values to make a more efficient study exploration. In total, 10 molecules, namely, MED6, MED8, MED10, MED17, MED19, MED20, MED21, MED22, MED24, and MED25, were included in the subsequent analysis.

### 3.3. Integrated Genetic, Coexpression, Protein-Protein Interaction, and Gene-Gene Interaction Analysis of MED Family Members in Patients with HCC

To investigate the role of the differentially expressed genes in the MED family in the genomic background, we used the cBioPortal web tool to examine the genetic alterations of the remaining members of the MED family. Our results showed that MED6, MED8, MED10, MED17, MED19, MED20, MED21, MED22, MED24, and MED25 were altered in 5%, 5%, 6%, 8%, 6%, 7%, 5%, 5%, 7%, and 7% of the HCC specimens, respectively (Figure 7(a)). In addition, we estimated the correlations of the differentially expressed molecules at the RNA level. The coexpression analysis revealed moderate correlations between MED8 and MED19, between MED17 and MED21, and between MED22 and MED25 (Figure 7(b)). To investigate the interactions of the molecules of interest at the protein level, we performed a protein-protein interaction network analysis on the STRING website. We identified 10 nodes and 45 edges in the protein-protein interaction network, with the highest combined score between MED10 and MED17 (Figure 7(c)). Functional analysis of these proteins revealed that strong bonds mediated the regulation of RNA polymerase II transcription-related mechanisms. In addition, we used the GeneMANIA web tool to further elucidate the potential functions of the proteins of interest. The results showed that the top three associated functional changes resided in the mediator complex, transcription initiation from the RNA polymerase II promoter, and initiation of DNA-templated transcription (Figure 7(d)). Given that similar genes may have similar functions, we extracted the top 100 genes that were most similar to the genes of interest on the GEPIA website (Supplementary Table 1).

### 3.4. Functional Enrichment Analysis of the MED Family in Patients with HCC

To further investigate the roles of the MED molecules of interest and the neighbouring genes, the online web tool Metascape was subsequently used to annotate their functions.  Figure 8(a) shows the GO/KEGG terms with the top 20 enriched functions. We found that these similar genes were mainly enriched in the nucleobase-containing compound catabolic process, regulation of chromosome organisation, and transcriptional regulation by TP53. Moreover, the nucleobase-containing compound catabolic process, transcriptional regulation by TP53, DNA repair, RNA splicing via transesterification reactions with bulged adenosine as nucleophile, ribonucleoprotein complex biogenesis, ncRNA metabolic process, regulation of translational initiation, nuclear-transcribed mRNA catabolic process, P53 downstream pathway, regulation of the DNA metabolic process, regulation of the small molecule metabolic process, positive regulation of protein ubiquitination, and regulation of glucose import were associated with the carcinogenesis and progression of HCC. Furthermore, the metabolic process, regulation of the biological process, negative regulation of the biological process, cellular component organisation and biogenesis, response to stimulus, positive regulation of the biological process, signalling, developmental process, multiorganism process, and localisation were the top 10 highly enriched items in the biological process module. To better elucidate the role of the MED family at the protein level, we constructed a protein-protein interaction network with the mCODE module discriminating the subtype function in detail (Figure 8(b)). A full list of the mCODE modules is presented in Supplementary Table 2. We selected the top 1 mCODE module with the highest predicted score. We found that the biological function was enriched in the RNA splicing via transesterification reactions with bulged adenosine as nucleophile, mRNA splicing via spliceosome, and RNA splicing via transesterification reactions.

### 3.5. Immune Cell Infiltration of the MED Family in Patients with HCC

Recently, great focus pivoted around the correlation between the MED family and the immune repertoires [11, 21, 22], which showed a stupendous potential for immune therapy. Accordingly, we conducted a systematic analysis of immune infiltrates with members of interest of the MED family by using the online database TIMER. The gene module was used to examine the correlation between the expression levels of the members of interest of the MED family, immune infiltration level, and immune cell type. We found that the expression levels of all the members of interest of the MED family, namely, MED6, MED8, MED10, MED17, MED19, MED20, MED21, MED22, MED24, and MED25, were significantly (*p* < 0.05) and positively associated with all types of immune cells, namely, B cells, CD8^+^ T cells, CD4^+^ T cells, macrophages, neutrophils, and dendritic cells (Figures 9(a)–9(j)). We found that MED20, MED24, and MED25 positively correlated with tumour purity (Figures 9(f), 9(i), and 9(j), respectively). To examine the clinical relevance of the members of interest of the MED family and tumour immune subsets, we used the “survival” module in TIMER to examine the prognostic value of the MED family. The log-rank test revealed that the expression levels of MED6, MED8, MED10, MED17, MED19, MED20, and MED22 could significantly (*p* < 0.05) discriminate patient survival (Figure 10). Moreover, we established the Cox proportional hazard model to adjust for confounding factors. Only B cell (*p* = 0.021) and MED8 (*p* = 0.034) independently predicted patient survival after eliminating confounders from CD8^+^ T cells, CD4^+^ T cells, macrophages, neutrophils, dendritic cells, MED6, MED10, MED17, MED19, MED20, MED21, MED22, MED24, and MED25 (Supplementary Table 3). Next, we determined the correlation between the somatic CNAs of the members of interest of the MED molecules and the abundance of immune infiltrates (Figure 11). We found that the arm-level deletion of MED6 significantly correlated with the macrophage infiltration level (*p* < 0.05; Figure 11(a)). The arm-level deletion of MED8, arm-level gain and high amplification of MED20, and arm-level gain of MED22 significantly correlated with the neutrophil cell infiltration level (*p* < 0.05, *p* < 0.05, *p* < 0.01, and *p* < 0.05, respectively; Figures 11(b), 11(f), and 11(h), respectively). The arm-level gain of MED10 and arm-level deletion of MED25 significantly correlated with CD4+ T cells (*p* < 0.05 and *p* < 0.05, respectively; Figures 11(c) and 11(j), respectively). Arm-level deletion of MED8, arm-level deletion of MED21, and high amplification of MED24 significantly correlated with CD8+ T cells (*p* < 0.01, *p* < 0.05, and *p* < 0.05, respectively; Figures 11(b), 11(g), and 11(i), respectively). The high amplification of MED20 and arm-level deletion of MED21 significantly correlated with B cells (*p* < 0.05 and *p* < 0.05, respectively; Figures 11(f) and 11(g), respectively).

## 4. Discussion

The MED family was initially examined for its transcriptional regulation activity since its discovery and involvement in multiple cancers in terms of its aberrant function in genomic mutation and transcription levels. The microenvironment in HCC is characterised by severe immunosuppression or exhaustion [23]. These unique tumour microenvironment characteristics in HCC indicate the promising therapeutic potential of immune therapy to overcome the relatively immunosuppressive tumour microenvironment before exhaustion. Currently, accumulating evidence shows the essential role of the MED family in the immune system, mediating the carcinogenesis and progression of diverse cancers [11, 12]. Given the immune regulatory characteristics of the MED family, we assumed that the MED family may possess therapeutic and prognostic values in patients with HCC.

In this study, we first examined the expression patterns of the MED family members in HCC with qualitative and quantitative methods. Our results showed a prevailing aberrant high expression pattern in all members of the MED family in HCC tumours compared with normal tissues. Moreover, we found that the expression levels of MED1, MED6, MED8, MED10 MED12, MED15, MED17, MED19, MED20, MED21, MED22, MED23, MED24, MED25, MED26, and MED27 significantly correlated with pathological stage. The patients with HCC who had high expression levels of MED6, MED8, MED10, MED17, MED19, MED20, MED21, MED22, MED24, and MED25 were significantly associated with worse prognosis in terms of the key factors, OS and DFS. These data suggest the essential role and clinical prognostic value of the MED family in HCC. Tsang et al. studied the aberrant super-enhancer landscape in HCC and found that the frequently overexpressed MED1 conferred worse OS and DFS in patients with HCC [24]. Similarly, Wang et al. reported that the MED15 expression level was an independent prognostic factor of OS in patients with HCC but was not an indicator of DFS [25]. Moreover, Guo et al. showed a frequently upregulated expression pattern of MED23, consistent with our discovery of the high expression patterns of all members of the MED family [26]. However, the integrated analysis of the prognostic value of the MED family in patients with HCC is limited.

To provide a thorough understanding of the molecular characteristics of the MED family, we conducted a systemic analysis of the MED molecules of interest in HCC. We found that genetic alteration events prevailed among the MED family members in the patients with HCC. Coexpression analysis revealed a moderate correlation with the differentially expressed MED molecules at the RNA level, consistent with the relatively tight protein-protein interaction, which suggested a direct synergistic role of the MED family in the carcinogenesis and progression of HCC.

As similar genes may have similar functions, we conducted a functional enrichment analysis of members of interest of the MED family with the top 100 most similar genes using GO/KEGG enrichment items. As expected, our results showed that these genes were enriched in carcinogenesis- and progression-related functions such as the transcriptional regulation by TP53 and ribonucleoprotein complex biogenesis. TP53, a frequently mutated tumour suppressor gene widely investigated in HCC, plays a key role in regulating the cell cycle, proliferation, apoptosis, and genomic integrity [27, 28]. Moreover, a prior report indicated that heterogeneous nuclear ribonucleoprotein A1 might be engaged in tumour formation via the EGFR signalling pathway in HBV-related HCC. In short, these data suggest that the MED family members play a significant role in HCC development and are potential therapeutic targets.

Moreover, we evaluated the immune characteristics of the MED family given the significant correlation between the MED family and the immune repertoires. In our study, we found a significant positive association between all MED family members of interest and all types of immune cells, namely, B cells, CD8^+^ T cells, CD4^+^ T cells, macrophages, neutrophils, and dendritic cells. This suggests that the MED family members might be promising biomarkers for the prediction of response to immune therapy. In addition, we demonstrated that MED8 could independently predict patient survival, indicating that MED8 might be a prognostic biomarker of HCC. However, further clinical trials are warranted to test the reliability of the prognostic performance of MED8 in HCC cases. Furthermore, we found a significant correlation between the somatic CNAs of the MED molecules and the abundance of immune infiltrates. Taken together, the MED family members are not only prognostic biomarkers but also possible participants in immune regulation.

Several caveats are worth underscoring regarding the limitations of our study. First, our data analysis was conducted using a single database (TCGA) without external comparison, which diminished the reliability of our results. Moreover, our analysis design was mainly based on the genome and transcriptome. However, a systematic analysis integrating proteomic data may provide new insight into the clinical value of the MED family in the diagnosis and treatment of patients with HCC. Moreover, additional studies *in vitro* or *in vivo* are warranted to confirm the aforementioned results.

## 5. Conclusion

In summary, our study delineates a thorough landscape to investigate the therapeutic and prognostic potentials of the MED family. With the feature of immune regulation, the MED family members are promising biomarkers, which yielded encouraging results for the development of immunotherapeutic drugs and construction of a prognostic stratification model. Further investigation of how the MED family is involved in modulating immune interactions, especially in HCC cases with TP53 mutation, given the aforementioned function annotation, will be interesting. Genes in the MED family are promising targets of HCC immune therapy.

## Figures and Tables

**Figure 1:** Pancancer analysis of MED family expression at RNA level. The numbers of unique significant analysis of upregulated expression (red) and downregulated expression (blue) of MED family at the transcriptional level were presented using the ONCOMINE web tool. MED: mediator complex.

**Figure 2:** Expression pattern of MED family in HCC. All of the molecules in MED family (a–g) showed an aberrantly high expression pattern in HCC tumours regarding normal tissue analysed quantitatively at the RNA level using the UALCAN website. The *p* value thresholds were set at 0.05. HCC: hepatocellular carcinoma; MED: mediator complex.

**Figure 3:** Comprehensive qualitative analysis of expression patterns of MED family in HCC. This figure shows that the relative expression of MED 16 was the highest scored at 5.2 while MED 26 scored 2 as the lowest counterpart. HCC: hepatocellular carcinoma; MED: mediator complex.

**Figure 4:** Correlation analysis within MED family and pathological stage of HCC cases: (a) MED1, MED6, and MED8; (b) MED10 and MED12; (c) MED15 and MED17; (d) MED19, MED20, MED21, MED22, and MED23; and (e) MED24, MED25, MED26, and MED27 were significantly correlated with the pathological stage of HCC conducted in the GEPIA website. The *p* value thresholds were set at 0.05. HCC: hepatocellular carcinoma; MED: mediator complex.

**Figure 5:** Kaplan–Meier estimates the prognostic value of MED family in OS. Kaplan-Meier survival curve of (a) MED1, (b) MED6, (c) MED8, (d) MED10, (e) MED12, (f) MED15, (g) MED17, (h) MED19, (i) MED20, (j) MED21, (k) MED22, (l) MED23, (m) MED24, (n) MED25, (o) MED26, and (p) MED27 for OS in HCC cases. The log-rank *p* value thresholds were set at 0.05. HCC: hepatocellular carcinoma; MED: mediator complex; OS: overall survival.

**Figure 6:** Kaplan–Meier estimates the prognostic value of MED family in DFS. Kaplan-Meier survival curve of (a) MED1, (b) MED6, (c) MED8, (d) MED10, (e) MED12, (f) MED15, (g) MED17, (h) MED19, (i) MED20, (j) MED21, (k) MED22, (l) MED23, (m) MED24, (n) MED25, (o) MED26, and (p) MED27 for DFS in HCC cases. The log-rank *p* value thresholds were set at 0.05. HCC: hepatocellular carcinoma; MED: mediator complex; DFS: disease-free survival.

**Figure 7:** Systemic analysis of genetic alteration, coexpression correlation and protein–protein interaction analyses of MED family in HCC cases. (a) Genetic alterations of MED family in HCC cases. (b) Correlation heat map of coexpression of MED family in HCC. (c, d) Protein–protein interaction network of MED family performed in GeneMANIA and STRING. HCC: hepatocellular carcinoma; MED: mediator complex.

**Figure 8:** Functional annotation of interested MED family and top 100 most similar genes in HCC cases. (a) GO-BP/CC/MF and KEGG pathway analyses presented in bar plot (top 20). BP: biological process; CC: cellular component; HCC: hepatocellular carcinoma; MED: mediator complex; MF: molecular function.

**Figure 9:** Correlation analysis of interested MED family and immune cell infiltration. The correlation within immune cell infiltration and transcriptional expression of (a) MED6, (b) MED8, (c) MED10, (d) MED17, (e) MED19, (f) MED20, (g) MED21, (h) MED22, (i) MED24, and (j) MED25 in HCC cases. HCC: hepatocellular carcinoma; MED: mediator complex.

**Figure 10:** Clinical prognostic value of interested MED family and tumour immune subsets. Kaplan-Meier survival curve of MED family and immune cell in HCC cases. The log-rank *p* value thresholds were set at 0.05. Log-rank *p* value < 0.001 was presented as log − rank *p* value = 0. HCC: hepatocellular carcinoma; MED: mediator complex.

**Figure 11:** Correlation analysis of somatic CNA of interested MED family and immune infiltration. The correlation within immune cell infiltration and somatic CNA of (a) MED6, (b) MED8, (c) MED10, (d) MED17, (e) MED19, (f) MED20, (g) MED21, (h) MED22, (i) MED24, and (j) MED25 in HCC cases. ^∗^*p* < 0.05, ^∗∗^*p* < 0.01. CNA: copy number aberration; HCC: hepatocellular carcinoma; MED: mediator complex; MF: molecular function.

## Data Availability

The data used to support the findings of this study are included within the article.

## Additional Points

*Code Availability*. This article does not contain any code to conduct the research.

## Supplementary Materials

Supplementary Materials Supplement Table 1: the top 100 genes that were most similar to the genes of interest on the GEPIA website. Supplement Table 2: the full list of mCODE for protein-protein interaction network. Supplement Table 3: construction of a multifactor Cox risk proportional model.
